The article "Fproi-GAN with Fused Regional Features for the Synthesis of High-Quality Paired Medical Images" was published in 2021. Journal: J Healthc Eng.

# Fp^roi^-GAN with Fused Regional Features for the Synthesis of High-Quality Paired Medical Images

**DOI:** 10.1155/2021/6678031

**Published:** 2021-04-26

**Authors:** Jiale Dong, Caiwei Liu, Panpan Man, Guohua Zhao, Yaping Wu, Yusong Lin

**Affiliations:** ^1^School of Information Engineering, Zhengzhou University, Zhengzhou 450001, China; ^2^Collaborative Innovation Center for Internet Healthcare, Zhengzhou University, Zhengzhou 450052, China; ^3^Department of Medical Imaging, Henan Provincial People's Hospital, Zhengzhou 450003, China; ^4^School of Software, Zhengzhou University, Zhengzhou 450002, China; ^5^Hanwei IoT Institute, Zhengzhou University, Zhengzhou 450002, China

## Abstract

The use of medical image synthesis with generative adversarial networks (GAN) is effective for expanding medical samples. The structural consistency between the synthesized and actual image is a key indicator of the quality of the synthesized image, and the region of interest (ROI) of the synthesized image is related to its usability, and these parameters are the two key issues in image synthesis. In this paper, the fusion-ROI patch GAN (Fp^roi^-GAN) model was constructed by incorporating a priori regional feature based on the two-stage cycle consistency mechanism of cycleGAN. This model has improved the tissue contrast of ROI and achieved the pairwise synthesis of high-quality medical images and their corresponding ROIs. The quantitative evaluation results in two publicly available datasets, INbreast and BRATS 2017, show that the synthesized ROI images have a DICE coefficient of 0.981 ± 0.11 and a Hausdorff distance of 4.21 ± 2.84 relative to the original images. The classification experimental results show that the synthesized images can effectively assist in the training of machine learning models, improve the generalization performance of prediction models, and improve the classification accuracy by 4% and sensitivity by 5.3% compared with the cycleGAN method. Hence, the paired medical images synthesized using Fp^roi^-GAN have high quality and structural consistency with real medical images.

## 1. Introduction

Medical imaging is a clinically important noninvasive diagnostic method; imaging specialists can diagnose breast cancer or precancer through mammography images [1]. With the development of deep learning technology, medical image synthesis [2, 3], classification [4], and segmentation [5] based on deep learning have become topical issues in medical research. Deep neural networks usually require a large number of training samples, and the size of medical image data is usually small because of the high collection cost, thus limiting the application of deep learning models for medical images [6]. Generative adversarial networks [7] usually learn feature mappings from source modality to target modality by constructing generators and discriminators that can be used to synthesize medical images and thus expand training samples [8, 9]. However, the gradient disappearance, pattern collapse, and structural consistency problems between real and synthetic images in the current GAN research process seriously affect the quality of synthetic images [3]. In addition, the region of interest (ROI) of medical images is a key factor in aiding imaging research and is often used in training medical image segmentation tasks. However, we found that the synthesis of the ROI has rarely been studied [10, 11]. Thus, in the present study, we focused on the synthesis of high-quality medical images and their ROI images.

Nie et al. [12] were the first to propose a generative adversarial model using a fully convolutional neural network as a generator that implements the conversion between MRI and CT images of brain tumor images. The 3D-based fully convolutional neural network proposed in this paper well solves the problem of discontinuity across slices in 2D neural networks, and the method improves the quality of the generated images by calculating the gradient difference of the images as a loss function. The experimental results show that the method proposed in this paper can effectively predict CT images from MRI images, which is an early research and exploration of generative adversarial networks in the field of medical image synthesis. Guibas et al. [13] propose a novel pipeline model based on generative adversarial networks for the current medical images that are not easily accessible. The model proposed in this paper consists of Stage-I GAN and Stage-II GAN, which enables the generation of higher quality images by enhancing the learning of mask image features of images. In addition, John et al. created an online synthetic medical image database called SynthMed, while again demonstrating the feasibility of GAN-based synthesis of medical images. In addition, Chartsias et al. [8] proposed a multi-input, multi-output fully convolutional neural network for MRI synthesis, which embeds all input modalities into a shared potential space and converts the shared features into target output modalities by learning the potential space mapping through a decoder. Although this method can achieve multimodal output, the generated images are adulterated with redundant information. Wolterink et al. [9] used cycleGAN to learn the mapping of source modality to target modality through adversarial loss, resulting in synthetic CT images that are similar to the real CT images. Considering the lack of direct constraints between the real CT images and the synthesized CT images, this approach still cannot guarantee the structural consistency between the synthesized and the input images. Kang et al. [14] proposed a conditional GAN to improve model estimation and quantitatively evaluate the resulting images, but this approach resulted in uneven quality across domains of the synthesized images. Huang et al. [15] synthesized glioma images by using the WEENIE model, which uses a priori information instead of noise as input to the model, but the consistency of the synthesized images with the real images needs to be improved.

In the study of GAN-based generative models, the structural consistency between the real and synthetic images usually affects the quality of the synthetic images [3]. To improve the structural inconsistency between the real and synthesized image during image synthesis and synthesize the ROI of the image, we proposed a new method for synthesizing paired medical images based on cycleGAN. The method incorporates regional a priori features on the basis of cycleGAN two-stage cycle consistency to achieve high-quality medical images and their ROI synthesis. In the medical image synthesis process, the first stage model implements feature mapping from the medical image domain to the ROI domain and targets the learning contrast features of ROI and non-ROI tissues. The second stage network reduces the ROI domain to the medical image domain to synthesize medical images. By contrast, in the synthesis process of ROI, the input ROI image is first reduced to a medical image, and then a high-quality ROI image is synthesized based on the regional contrast of the medical image. The two-stage synthesis process is implemented through the cycle consistency function of cycleGAN [16]. In this paper, we validated the quality of the synthesized images by using two publicly available datasets, where the benign data of the INbreast dataset has no corresponding ROI images. Then, we quantitatively analyzed the synthesis results from various metrics only. The results show that our proposed method effectively improves the structural consistency between the synthesized and real image, and the quality of the synthesized image is better than several recent popular models. In addition, we have verified that the images synthesized in this paper can improve the classification performance of the prediction model in the brain glioma classification experiment. The experimental results demonstrate that the method in this paper can effectively generate high-quality paired medical images, which will bring new solutions for medical disease research where it is difficult to obtain data.

The contribution of this work is summarized as follows.

1. We proposed a new synthesis method for the synthesis of paired medical images on the cycle consistency mechanism of cycleGAN and called it Fp^roi^-GAN
2. To improve the quality of the synthesized images, this paper assists the generative model to learn ROI and non-ROI organizational features by supplementing a priori regional features
3. Fp^roi^-GAN proved its effectiveness on two experimental datasets, and the experimental results show that our method can effectively improve the structural consistency of synthesized images with real images and outperform many popular image synthesis methods

## 2. Materials and Methods

### 2.1. Dataset

INbreast [17, 18] contains 303 normal (no mass) mammograms and 107 pairs of mammograms, including mass data and corresponding ROI images. Considering that training requires paired data, only 107 pairs of images containing masses were finally selected as the experimental data and then preprocessed. The mammograms had a resolution of 3,328 × 4,084 pixels or 2,560 × 3,328 pixels, and the images were stored in dicom format. We first cropped the original images according to the provided lesion areas, and the cropped images to 256 × 256 were converted into PNG format, as shown in Figure 1(a). The processed paired data were divided into training and test sets in a ratio of 7 : 3, and the image intensity was linearly normalized to [0,1] by using maximum normalization. Subsequently, the influence of data irregularity on the experimental results was eliminated, and the network was accelerated to determine the optimal solution.

The BRATS 2017 [19, 20] dataset contains 285 medical images and their corresponding ROI images from four sequences, Tl-weighted (T1), Tl-weighted and contrast-enhanced (T1ce), T2-weighted (T2), and FLAIR, including 210 high-grade gliomas (HGG) and 75 low-grade gliomas (LGG), with image sizes of 240 × 240 × 155 voxels. T2 sequences were selected as the experimental data, and the 90th and 100th layer slices of the HGG images (the middle layer contains more brain image information relative to the edge of the voxel images) and the corresponding ROI slices were extracted first. Similarly, the 90th, 95th, 100th, and 105th layer slices of LGG images and the corresponding ROI slices were extracted, and each of the 272 pairs of HGG and LGG images were collected, as shown in Figure 1(b). Finally, all images were adjusted to 256 × 256 pixels. The two small datasets, HGG and LGG, were normalized according to INbreast's partitioning and processing method.

### 2.2. Methods

To enable the network learn the contrast information of ROI and non-ROI tissues, we improved the cycleGAN model and proposed a pairwise image synthesis method that incorporates regional features.  Figure 2 shows the flowchart of the model, where the input of the network is the medical image and its corresponding ROI. Before the network started training, the medical image matrix was first multiplied with its ROI image matrix to obtain the regional image containing only the tumor. Then, we designed a regional feature extraction block (RFB) to extract the semantic features of regional images and fuse the extracted regional features with medical images as the input of source domain *X* and ROI as the input of target domain *Y*. During network training, the model discriminates between ROI and non-ROI organizational features by learning the mapping of domain *X* to domain *Y*. The a priori regional features enhance the learning process and then reduces domain *Y* to domain *X* to synthesize medical images. ROI synthesis first reduces the mapping of domain *Y* to domain *X* and synthesizes high-quality ROI images based on the mapping of domain *X* to domain *Y*. Figure 2(c) shows the synthesis of medical images, and the process can be represented as: *x*⟶*G*(*x*)⟶*F*(*G*(*x*)) ≈ *x* as shown in (i); similarly, the synthesis process of ROI can be represented as: *y*⟶*F*(*y*)⟶*G*(*F*(*y*)) ≈ *y*, as shown in (ii). The model proposed in this paper is composed of two generators, namely, *G* and *F*, and two discriminators, namely, *D*_*x*_ and *D*_*y*_.

#### 2.2.1. Regional Feature Extraction

First, the medical image was multiplied with the ROI matrix to obtain the regional image, and the operation steps are shown in Figure 2(a). We designed the RFB for extracting high-level semantic features of the region image, and its structure is shown in Figure 3. The feature extraction block is a simple convolutional neural network consisting of two mirror fill layers, three convolutional layers, and one deconvolutional layer. In the network, the operational details of the three convolutional layers are zoomed into the right side of Figure 3, where the convolutional details include convolution, instance normalization, and activation operations. The feature map output after the RFB is fused with the medical image as the input of domain *X*.

#### 2.2.2. Network Architecture

The Fp^roi^-GAN model consists of two generators and two discriminators, where the structures of the generators *G* and *F* are shown in Figure 4. The generator consists of four convolutional layers, two fusion layers, and two deconvolutional layers, and the operation details of each convolutional layer include convolution, instance normalization, and activation operations. To extract each pixel in the fused image, the generator first performs a 3 × 3 mirror fill of the image, and the feature map size is filled from 256 × 256 pixels to 262 × 262 pixels after filling. After three convolution processes, a 128-dimensional 64 × 64 feature map is obtained. The convolution aims to downsample the image and extracts its structural features, where the details of the three convolution layer operations are zoomed into the corresponding color boxes on both sides. In addition, we added two fusion layers to the generator to preserve the low-level image information. Finally, two deconvolution layers restore the image to its initial size and complete the image synthesis.

The inputs of the discriminator *D*_*x*_ include real and synthetic medical images, while the inputs of the discriminator *D*_*y*_ include synthetic and real ROI images. The discriminator consists of four convolutional layers, flatten layer, dense layer, and sigmoid activation layer. The convolved image is flattened by the flatten layer, and the dense layer reduces the features to one dimension. Finally, the sigmoid function determines whether the image is synthetic or real, and the details of the discriminator layers are depicted in Figure 5. The discriminator is executed immediately after the output of the generator.

#### 2.2.3. Training Loss

The loss functions used in the synthesis of the images include the traditional adversarial [7] and cycle consistency loss [16]. The model uses adversarial loss as the mapping function. The mapping function *G* : *X*⟶*Y* and its discriminator *D*_*Y*_ are expressed in (1) as follows:

(1) $$\begin{array}{c} {ℒ}_{\text{GAN}}\left(G,D_{Y},X,Y\right)=E_{y∼P_{\text{data}}\left(y\right)}\left[\log\;\;D_{Y}\left(y\right)\right]+E_{x∼P_{\text{data}}\left(x\right)}\left[\log\left(1-D_{Y}\left(G\left(x\right)\right)\right)\right], \end{array}$$

where *G*(*x*) generates an image similar to the *Y* domain, and *D*_*Y*_ distinguishes between the synthesized sample and the real sample. In this process, *G*(*x*) aims to distinguish between information from ROI and non-ROI tissue, resulting in subsequent *F*(*G*(*x*)) restoration process. *G* aims to minimize this objective against an adversary *D*_*Y*_ that tries to maximize it, in which min_*G*_max_*D*_*Y*__ℒ_GAN_(*G*, *D*_*Y*_, *X*, *Y*). Similarly, in the restoration process of *F*(*G*(*x*)), a similar mapping function*F* : *Y*⟶*X* learns the mapping from the ROI image to the medical image, in which min_*F*_max_*D*_*X*__ℒ_GAN_(*F*, *D*_*X*_, *Y*, *X*), where *D*_*X*_ represents its discriminator.

Traditional adversarial losses can only intermittently learn the mapping function from domain *X* to domain *Y* or vice versa. To constrain the consistency of the real image with the synthetic image, we used a cycle consistency loss function in the model to enhance the reduction process. In Figure 2(c), *x*⟶*G*(*x*)⟶*F*(*G*(*x*)) ≈ *x* constrains the synthesis process of the medical image, while *y*⟶*F*(*y*)⟶*G*(*F*(*y*)) ≈ *y* constrains the synthesis process of the ROI image. These two components constitute the cycle consistency loss, as shown in the following:

(2) $$\begin{array}{c} {ℒ}_{\text{cyc}}\left(G,F\right)=E_{x∼P_{\text{data}}\left(x\right)}\left[{\left\|F\left(G\left(x\right)-x\right)\right\|}_{1}\right]+E_{y∼P_{\text{data}}\left(y\right)}\left[{\left\|G\left(F\left(y\right)-y\right)\right\|}_{1}\right]. \end{array}$$

### 2.3. Evaluation Measures

The peak signal-to-noise ratio (PSNR) [21], structural similarity (SSIM) [22], and multiscale structural similarity (MS-SSIM) [23] were used for the quantitative evaluation of the synthesized medical images. Dice coefficient and Hausdorff distance were used for the quantitative evaluation of the synthesized ROI images. Given the original input and synthetic images, the PSNR can be defined as follows:

(3) $$\begin{array}{c} \text{PSNR}\left(x,F\left(G\left(x\right)\right)\right)=10{\text{log}}_{10}\frac{{\text{MAX}}_{\text{range}}^{2}\left(x,F\left(G\left(x\right)\right)\right)}{N_{\text{voxel}}^{-1}{\left\|x-F\left(G\left(x\right)\right)\right\|}_{2}^{2}}\;, \end{array}$$

where MAX_range_(*x*, *F*(*G*(*x*))) represents the maximum number of pixels for *x* and *F*(*G*(*x*)) images, and *N*_voxel_ represents the total number of pixels for *x* or *F*(*G*(*x*)). The higher the PSNR value, the better the synthesis performance. SSIM was used to measure three metrics of image brightness, contrast, and structure, which can be expressed as follows:

(4) $$\begin{array}{c} \text{SSIM}\left(x,F\left(G\left(x\right)\right)\right)=\frac{\left(2\mu_{x}\mu_{F\left(G\left(x\right)\right)}+c_{1}\right)\left(2\sigma_{xF\left(G\left(x\right)\right)}+c_{2}\right)}{\left(\mu_{x}^{2}+\mu_{F\left(G\left(x\right)\right)}^{2}+c_{1}\right)\left(\sigma_{x}^{2}+\sigma_{F\left(G\left(x\right)\right)}^{2}+c_{2}\right)}, \end{array}$$

where *μ* and *σ*^2^ denote the mean and variance of the image, respectively, and *σ*_*xF*(*G*(*x*))_ denotes the covariance of *x* and *F*(*G*(*x*)). The closer the SSIM is to 1, the higher the structural similarity is. The larger MS-SSIM values represent a better synthesis performance [24]. Dice coefficients [25, 26] are often used to represent the performance of the synthesized ROI image based on the ROI image *y* and the synthesized ROI images *G*(*F*(*y*)) as follows:

(5) $$\begin{array}{c} \text{Dice}\left(y,G\left(F\left(y\right)\right)\right)=\frac{2\left|y\cap G\left(F\left(y\right)\right)\right|}{\left|y\right|+\left|G\left(F\left(y\right)\right)\right|}. \end{array}$$

The Hausdorff distance [27], a complement to the Dice evaluation metric, can be expressed as follows:

(6) $$\begin{array}{c} \text{Hausdorff}\left(y,G\left(F\left(y\right)\right)\right)=\text{max}\left({\text{max}}_{y\in y}\left(\text{min}\left(d\left(y,G\left(F\left(y\right)\right)\right)\right)\right),{\text{max}}_{G\left(F\left(y\right)\right)\in G\left(F\left(y\right)\right)}\left(\text{min}\left(d\left(y,G\left(F\left(y\right)\right)\right)\right)\right)\right), \end{array}$$

where *d* represents the Euclidean distance.

## 3. Results and Discussion

Our network implementation was based on the PyTorch framework. All experiments were performed on a 12-core Intel Xeon 3.7 GHz CPU and GeForce RTX 2080 (8 GB) by using the Ubuntu 18.04 operating system. All figures were plotted on a computer with Windows 10 (8 GB) operating system. During the synthesis task, all models were trained for 300 epochs, where the trained models used the Adam optimizer [28] with default parameters, and the learning rate was set to 0.0002.

### 3.1. Results of the INbreast Dataset

This subsection provides a comparison of three commonly used synthesis models, namely, DCGAN [11], Pix2Pix [15], and cycleGAN [16].  Table 1 evaluates the whole and tumor domains of the synthesized images, and Table 2 compares the synthesis results of ROI images. Tables 1 and 2 compare the differences between Fp^roi^-GAN and the other methods using paired-samples *T*-tests [29], and the underline indicates a significant difference between Fp^roi^-GAN and the other methods at a significance level of 0.05. Based on the experimental results in Table 1, the Fp^roi^-GAN image synthesis method achieved the highest results for the three evaluation metrics, whereas the DCGAN synthesized image results were the lowest. Based on the quantitative analysis results of the whole image domain, the Fp^roi^-GAN values were 0.832, 0.053, and 0.016 higher than those of the cycleGAN method in the three evaluation metrics of PSNR, SSIM, and MS-SSIM, respectively, and 1.813, 0.113, and 0.056 higher than the DCGAN, respectively. In the tumor domain, the Fp^roi^-GAN values were 3.657, 0.085, and 0.042 higher than those of the cycleGAN method in the three evaluation metrics of PSNR, SSIM, and MS-SSIM, respectively, and 4.911, 0.095, and 0.052 higher than the DCGAN method, respectively. Fp^roi^-GAN method was significantly improved relative to other synthesis methods in Table 1. Based on the experimental results in Table 2, Fp^roi^-GAN obtained the highest DICE coefficient, which is 0.154 higher than DCGAN, and the lowest evaluated value in Hausdorff Distance, which is 3.10 lower than DCGAN.  Figure 6 shows the visual performance of the four synthesis methods, and Fp^roi^-GAN performs closer to the original image in some detail positions.

### 3.2. Results of the BraTS 2017 Dataset

This subsection provides comparison with three commonly used synthetic models, such as DCGAN [11], Pix2Pix [15], and cycleGAN [16]. Tables 3 and 4 compare the differences between Fp^roi^-GAN and other methods by using paired-sample *t*-test [29], and the underline indicates that Fp^roi^-GAN is statistically significantly different from other methods at a significance level of 0.05. Based on the experimental results in Table 3, the quantitative analysis results of Fp^roi^-GAN in the HGG data for the whole image domain are higher than those of cycleGAN in PSNR, SSIM, and MS-SSIM by 0.604, 0.002, and 0.003, respectively, and by 9.135, 0.104, and 0.097, compared with DCGAN, respectively. In the tumor domain, the Fp^roi^-GAN values were higher than cycleGAN in PSNR, SSIM, and MS-SSIM by 6.236, 0.02, and 0.023, respectively, and 12.349, 0.094, and 0.083 higher than DCGAN method, respectively. The quantitative analysis results of Fp^roi^-GAN in LGG data in the whole image domain are 1.999, 0.006, and 0.008 higher than cycleGAN in the three evaluation metrics of PSNR, SSIM, and MS-SSIM, respectively, and 6.951, 0.069, and 0.066 higher than DCGAN, respectively. In the tumor domain, the Fp^roi^-GAN values were 11.248, 0.004, and 0.007 higher than cycleGAN and 14.631, 0.105, and 0.079 higher than DCGAN.

Based on the experimental results in Table 4, Fp^roi^-GAN in HGG data achieved the highest DICE coefficient, which is 0.128 higher than DCGAN, and the lowest evaluated value in Hausdorff distance, which is 3.44 lower than DCGAN. The DICE coefficient of Fp^roi^-GAN in LGG data part was higher than DCGAN by 0.101, and the Hausdorff distance was lower than DCGAN by 3.75.  Figure 7 shows the visual results of the four synthesis methods, in which the synthesis results of the tumor domain, as well as the results of the non-tumor domain, are compared, as shown in the medical images of LGG. III shows the results of the synthesized paired images in ITK-SNAP [30], and the results show that Fp^roi^-GAN method has less noise points than the other synthesis methods. The results of the image distribution of the four synthesis methods are compared in Figure 8, where the histogram indicates the distribution of the image grayscale and the trend of the image grayscale. The Fp^roi^-GAN method is always closer to the original image than the three other methods, both in terms of image distribution and trend of image grayscale.

In addition to the quantitative evaluation of the synthesized MR images, this paper supplements a glioma HGG and LGG classification experiment to verify the auxiliary effect of the synthesized MR images for the classification experiment. Considering that the INbreast dataset without mass data lacks corresponding ROI images, our synthesis method is not applicable, and the auxiliary effect on its dataset could not be verified in the classification. In the image synthesis experiments, the training set included 380 images, consisting of 190 HGG and LGG data, and the test set included 164 images, consisting of 82 HGG and LGG data. In the classification experiments, the data used for testing in the synthesis method were used as the training set with 164 images, the data used for training in the synthesis method were used as the test set with 380 images, and the data from each of the four groups synthesized images were added as comparison experiments, as shown in Table 5. Referring to article [31, 32] for the classification method, the first 500 features were extracted for each group of images by using the Resnet [33] network, followed by 30 features selected by the recursive feature elimination [34] with fivefold cross-validation, and the filtered features were classified using the kernel-based SVM algorithm [35]. The metrics used to assess the classification results include AUC, accuracy (Acc), sensitivity (Sen), and specificity (Spe), where AUC represents the area of the ROC curve and the other three metrics can be defined as (7)–(9):

(7) $$\begin{array}{c} \text{Acc}=\frac{\text{TP}+\text{TN}}{\text{TP}+\text{FP}+\text{TN}+\text{FN}}, \end{array}$$

(8) $$\begin{array}{c} \text{Sen}=\frac{\text{TP}}{\text{TP}+\text{FN}}, \end{array}$$

(9) $$\begin{array}{c} \text{Spe}=\frac{\text{TN}}{\text{FP}+\text{TN}}, \end{array}$$

where TP represents the number of samples, in which HGG was correctly predicted, TN represents the number of samples, in which LGG is correctly predicted, FN represents the number of samples, in which HGG is predicted as LGG, and FP represents the number of samples, in which LGG is predicted as HGG. The experimental results in Table 5 show that, by adding the images synthesized by our method for training the machine learning model, the prediction ability of the model was effectively improved, in which Fp^roi^-GAN achieved the best results in the four metrics, and our method achieved a high classification sensitivity of 0.913. The ROC of the classification experiments is shown in Figure 9.

### 3.3. Discussion

Currently, most image synthesis methods are in single-input, single-output mode, and the synthesis of ROI images is rarely studied. Our work utilizes the cycleGAN's cyclic consistency mechanism to solve the problem of structural inconsistency between real and synthetic images and improves the contrast information between ROI and non-ROI domains by incorporating regional features a priori, resulting in the synthesis of high-quality medical images as well as the corresponding ROI images. To evaluate the quality of the synthesized images, we compared several currently popular synthesis methods, such as DCGAN, Pix2Pix, and cycleGAN, and evaluated the synthesis results in terms of the whole image domain of the images and the tumor domain. The results show that the Fp^roi^-GAN method synthesized high-quality medical images on both datasets and achieved the best results in PSNR, SSIM, MS-SSIM, dice, and Hausdorff distance metrics. The poor quality of the DCGAN synthesized images may be due to the collapse of the model during training, and we found that the synthesized images of Pix2Pix and cycleGAN are not of high quality due to the low structural consistency of the model. In addition, the comparison results from the whole and tumor domain of the images showed that the tumor domain is more informative than the whole domain by incorporating regional features.

As shown in Figure 7, our synthesis method resulted in the least noise points in the medical image processing tool ITK-SNAP, but the images generated by DCGAN contain more noise points. Based on the image distribution and grayscale change trend in Figure 8, the proposed method is closest to the distribution of the original image. From the previously mentioned experimental evaluation results, the sets of experiments show that the method proposed in this paper is more likely to be applied in the near future research of medical images. At last, in the BRATS 2017 classification experiments, we supplemented the synthesized data into the training set to effectively assist the training of the machine learning model and improve the classification effect of the model, in which the highest classification accuracy was achieved by adding the data synthesized by the Fp^roi^-GAN method. Although many adversarial generation models have been proposed, the quality of the generated images has been an important goal for researchers to pay attention to, and in addition, whether the generated images can be used in recent studies is also a key concern for research. In this paper, our proposed method generates high-quality images and is validated in brain glioma classification experiments, which proximately illustrates the feasibility and superiority of our proposed generation method in the process of medical imaging research.

## 4. Conclusions

GAN is widely studied in the field of medical imaging, including cross-modal synthesis, super-resolution reconstruction, and medical image denoising. In this paper, we proposed the Fp^roi^-GAN method to synthesize paired medical images. Moreover, we validated the results of the synthesized images via quantitative analysis, image distribution comparison, and visual evaluation. In the BRATS experiment, we added a classification experiment to verify the effect of synthesized data on the classification experiment. The results show that the addition of synthetic images effectively assisted the training of the machine learning model and improved the classification performance of the prediction model. Although this paper does not further validate the impact of the synthesized ROI images on the segmentation problem, the quantitative analysis indicated that our method has higher quantitative evaluation results than the other synthesis methods. In the future, we will further determine the effect of synthetic images on tasks, such as medical image classification and segmentation.

## Figures and Tables

**Figure 1:** (a) Cropping of the INbreast. (b) Slices containing tumor regions were extracted from the 3D images of glioma; × indicates that images that do not contain tumor domains were excluded.

**Figure 2:** (a) Regional feature extraction method. (b) The base model is a like-cycleGAN model consisting of two generators and two discriminators. (c) Synthesis of paired images. (i) Process synthesis of medical images. (ii) Process synthesis of ROI images.

**Figure 3:** RFB architecture; the convolution process zoomed into the box on the right side corresponding to the dimension.

**Figure 4:** Generator architecture; the convolution details of the generator are zoomed into the boxes on both sides.

**Figure 5:** Discriminator architecture; Conv2D and LeakyReLU layers were applied to all Conv blocks.

**Figure 6:** Comparison of Fp^roi^-GAN with the three other synthesis methods on the INbreast dataset. (a) Input image. (b) DCGAN. (c) Pix2Pix. (d) cycleGAN. (e) Fp^roi^-GAN.

**Figure 7:** Comparison of Fp^roi^-GAN with the three other synthesis methods on the BRATS 2017 dataset, where III is the visual performance in ITK-SNAP. (a) Input image (HGG). (b) DCGAN. (c) Pix2Pix. (d) cycleGAN. (e) Fp^roi^-GAN. (f) Input image (LGG). (g) DCGAN. (h) Pix2Pix. (i) cycleGAN. (j) Fp^roi^-GAN.

**Figure 8:** Image distribution results and grayscale trends of the four synthesis methods under HGG and LGG, where Fp(roi)-GAN represents Fp^roi^-GAN. (a) HGG. (b) LGG.

**Figure 9:** ROC plot of the classification experiment. (a) BRATS 2017. (b) BRATS 2017 + DCGAN. (c) BRATS 2017 + Pix2Pix. (d) BRATS 2017 + cycleGAN. (e) BRATS 2017 + Fp^roi^-GAN.

**Table 1:** Quantitative evaluation of the INbreast dataset (mean ± standard deviation). We compared the measurements of the different synthesis methods over the whole image domain and the tumor domain at a significance level of 0.05, and the underline indicates that Fp^roi^-GAN is statistically significantly different from other methods.

Region	Methods	PSNR	SSIM	MS-SSIM
Whole image	DCGAN [11]	16.834 ± 3.28	0.769 ± 0.15	0.879 ± 0.21
	Pix2Pix [15]	17.398 ± 3.81	0.843 ± 0.13	0.923 ± 0.19
	cycleGAN [16]	17.815 ± 5.18	0.829 ± 0.17	0.919 ± 0.18
	**Fp** ^**roi**^ **-GAN**	**18.647** **±** **3.25**	**0.882** **±** **0.16**	**0.935** **±** **0.15**

Tumor region	DCGAN [11]	19.231 ± 7.43	0.872 ± 0.15	0.894 ± 0.23
	Pix2Pix [15]	21.811 ± 6.98	0.915 ± 0.11	0.902 ± 0.22
	cycleGAN [16]	20.485 ± 6.15	0.882 ± 0.07	0.904 ± 0.18
	**Fp** ^**roi**^ **-GAN**	**24.142** **±** **6.70**	**0.967** **±** **0.08**	**0.946** **±** **0.18**

**Table 2:** Results of the quantitative evaluation of the ROI images of the INbreast dataset (mean ± standard deviation) with a significance level of 0.05; the underline indicates that the Fp^roi^-GAN is statistically significantly different from other methods.

Methods	Dice coefficient	Hausdorff distance
DCGAN [11]	0.827 ± 0.25	7.31 ± 4.95
Pix2Pix [15]	0.945 ± 0.17	7.27 ± 4.18
cycleGAN [16]	0.952 ± 0.13	6.83 ± 3.38
**Fp** ^**roi**^ **-GAN**	**0.981** **±** **0.11**	**4.21** **±** **2.84**

**Table 3:** Results of the quantitative evaluation of the BRATS 2017 dataset (mean ± standard deviation), where we compare the measurements of the different synthesis methods over the whole image domain and the tumor domain at a significance level of 0.05, and the underline indicates that Fp^roi^-GAN is statistically significantly different from the other methods.

Data	Region	Methods	PSNR	SSIM	MS-SSIM
HGG	Whole image	DCGAN [11]	25.749 ± 3.49	0.882 ± 0.04	0.890 ± 0.05
		Pix2Pix [15]	28.938 ± 4.68	0.952 ± 0.03	0.956 ± 0.05
		cycleGAN [16]	34.280 ± 4.85	0.984 ± 0.02	0.984 ± 0.05
		**Fp** ^**roi**^ **-GAN**	**34.884** **±** **5.18**	**0.986** **±** **0.02**	**0.987** **±** **0.04**
	Tumor region	DCGAN [11]	29.539 ± 5.05	0.903 ± 0.02	0.910 ± 0.05
		Pix2Pix [15]	33.031 ± 5.99	0.951 ± 0.02	0.952 ± 0.04
		cycleGAN [16]	35.652 ± 5.97	0.977 ± 0.03	0.970 ± 0.04
		**Fp** ^**roi**^ **-GAN**	**41.888** **±** **6.06**	**0.997** **±** **0.004**	**0.993** **±** **0.03**

LGG	Whole image	DCGAN [11]	23.093 ± 4.71	0.895 ± 0.11	0.908 ± 0.06
		Pix2Pix [15]	25.912 ± 4.95	0.933 ± 0.09	0.945 ± 0.07
		cycleGAN [16]	28.045 ± 4.47	0.958 ± 0.08	0.966 ± 0.03
		**Fp** ^**roi**^ **-GAN**	**30.044** **±** **4.21**	**0.964** **±** **0.08**	**0.974** **±** **0.03**
	Tumor region	DCGAN [11]	25.809 ± 4.39	0.892 ± 0.09	0.911 ± 0.07
		Pix2Pix [15]	30.228 ± 5.28	0.939 ± 0.08	0.948 ± 0.07
		cycleGAN [16]	29.192 ± 7.22	0.993 ± 0.01	0.983 ± 0.06
		**Fp** ^**roi**^ **-GAN**	**40.440** **±** **7.51**	**0.997** **±** **0.02**	**0.990** **±** **0.03**

**Table 4:** Results of the quantitative evaluation of the ROI images of the BRATS 2017 dataset (mean ± standard deviation) with a significance level of 0.05; underline indicates that the Fp^roi^-GAN is statistically significantly different from other methods.

Data	Methods	Dice coefficient	Hausdorff distance
HGG	DCGAN [11]	0.808 ± 0.29	8.36 ± 5.66
	Pix2Pix [15]	0.876 ± 0.23	7.54 ± 5.90
	cycleGAN [16]	0.931 ± 0.18	5.15 ± 3.03
	**Fp** ^**roi**^ **-GAN**	**0.936** **±** **0.18**	**4.92** **±** **3.22**

LGG	DCGAN [11]	0.889 ± 0.26	7.83 ± 4.84
	Pix2Pix [15]	0.947 ± 0.23	6.25 ± 3.12
	cycleGAN [16]	0.984 ± 0.21	4.66 ± 2.33
	**Fp** ^**roi**^ **-GAN**	**0.990** **±** **0.25**	**4.08** **±** **2.79**

**Table 5:** Classification results.

Data	Methods	AUC	Acc	Sen	Spe
BRATS2017	Resnet + SVM	0.872	0.789	0.823	0.778
BRATS2017 + DCGAN		0.881	0.803	0.720	0.831
BRATS2017 + Pix2Pix		0.894	0.815	0.857	0.855
BRATS2017 + cycleGAN		0.928	0.855	0.910	0.843
BRATS2017 + **Fp**^**roi**^**-GAN**		**0.943**	**0.882**	**0.913**	**0.868**

## Data Availability

The datasets used in this paper are public dataset BRATS2017 and public dataset INbreast. BRATS2017 can be obtained through the following URL: https://www.med.upenn.edu/sbia/brats2017/data.html, and INbreast can be obtained through the following URL: http://medicalresearch.inescporto.pt/breastresearch.
